# *Salvadora persica*'s Biological Properties and Applications in Different Dental Specialties: A Narrative Review

**DOI:** 10.1155/2022/8667687

**Published:** 2022-05-22

**Authors:** Fahd Aljarbou, Abdulaziz Almobarak, Abdulaziz Binrayes, Hadi M. Alamri

**Affiliations:** ^1^Department of Restorative Dental Sciences, Division of Endodontics, College of Dentistry, King Saud University, Riyadh 11545, Saudi Arabia; ^2^Department of Prosthodontics, Division of Endodontics, College of Dentistry, King Saud University, Riyadh 11545, Saudi Arabia; ^3^Conservative Dental Sciences, College of Dentistry, Prince Sattam Bin Abdulaziz University, Alkharj 11942, Saudi Arabia

## Abstract

*Salvadora persica* is a tree that belongs to the salvadorecea family. It is also known as Miswak, which is a popular natural toothbrush that was used centuries ago in oral hygiene by Muslims in all parts of the world, especially in the Middle East. Numerous researchers highlighted the biological activity of this plant in medicine, dentistry, and pharmacology. The purpose of this article is to narratively review the biological properties of *Salvadora persica*. In addition, it expresses variant applications of this herb in different dental specialties. *Materials and Methods*. The search of the literature was based on PubMed, MEDLINE, and Google Scholar using keywords: *Salvadora persica*, *S. persica*, Miswak, Dentistry, and Dental. All relevant articles were reviewed to check if they would fit within the scope of this review, and then, the information was extracted. *Results*. Multiple biological effects of *S. persica* have been reported including antibacterial, antiviral, antifungal, antibiofilm, antioxidant, and even antiulcer effects. Dental effects were discussed and presented. *Conclusion.* The wide biological range of *Salvadora persica*'s effects is promising for dental and nondental fields and allows for an expanded clinical application that has otherwise not been discussed in the literature.

## 1. Introduction

Herbal medicine was considered at the periphery of medicine in the near past. Nowadays, it is gaining popularity as an alternative type of treatment or medical interference due to its effectiveness in treating various types of diseases. A growing interest in the use of natural products, especially those from plants, has been more obvious. Several reasons account for this interest in plant-derived drugs, including a vast number of chemically and biologically unscreened plants and a long history of traditional medicine, suggesting the safety and effectiveness of natural product use [1]. The plant kingdom possesses rich and unique resources for the development of new leads and drugs for widely different pharmacological targets. In fact, many medications that have been widely used were either extracted from herbs or contain herbal ingredients. However, most of the herbal medications used were chemically extracted in various ways rather than consisting of a whole plant. Generally, herbs are plants that have leaves and seeds and that lack woody stems. Medical herbs are those used for their various medical properties and therapeutical effects [2]. Phytotherapy alludes to the medical treatment of diseases using health-promoting plants [3]. Many plants with medical benefits have been investigated, such as echinacea, caraway, chamomile, myrrh, and *Salvadora persica*.

In dentistry, the use of herbs has been advocated for treating or preventing specific microorganisms that are the cause of most dental diseases. A systematic review by Karygianni et al. tested the activity of multiple herbs on common oral pathogens. *Azadirachta indica*, also known as the neem tree, had an effect on *Streptococcus* spp., while *Camellia sinesis* affected both *Streptococcus mutans* and *Streptococcus sobrinus*. In addition, *Coffea arabica* and *Mikania laevigata* showed activity against *Streptococcus* spp. *Vaccinium macrocarpon* had an effect on *Streptococcus* spp. and *Porphyromonas gingivalis*. The researchers affirmed the negative effect of *Salvadora persica* (*S. persica*) on the growth of *Porphyromonas gingivalis*, *Aggregatibacter actinomycetemcomitans*, and *Haemophilus influenzae* [4]. The latter herb has been our focus here due to its added value in dentistry.

*Salvadora persica* (*S. persica*) is a small, soft, light-yellow woody tree that branches to form a large leafy bush with a widely spreading crown, flexible branches, and green-yellow flowers, with a life span of 25 years. It grows in dry and desert areas, preferably with black and loamy soils, and can form up to 10% of the local vegetation in some natural habitats. Moreover, it is an evergreen perennial halophyte capable of growing under extreme conditions, from very dry environments to highly saline soils. It possesses high potential for economic value as a source of oil and medicinal compounds [5]. In desert areas, a high proportion of root to shoot perennials is seen. *S. persica* can be found as deep-rooted mesomorphic xerophytes and as facultative halophytes that are highly salt-tolerant. Extremely high salt concentrations can reduce shoot and leaf growth [6]. *S. persica* is frequently used in folk medicine. The name *Salvadora* was first proposed in 1749 by Dr. Laurent Garcin, who was a well-known traveler and plant collector. He created the name in homage to Juan Salvador Bosca from Barcelona. The name persica means “Persia,” which refers to the Persian culture [7]. It is widely used by several populations worldwide, more frequently by Muslims. This has attracted our attention with regard to carrying out phytochemical and biological studies on the extracts and isolated compounds from *S. persica* as part of efforts to explore therapeutic agents from local plants [8]. Locally, it has great popularity, as shown in the survey by Sher et al. in 2011 [9]. They evaluated different parts of Saudi Arabia to obtain information about the folklore-related uses and the knowledge that local people and traditional healers held about this popular plant. Based on the results, it was concluded that *S. persica* has a versatile medicinal use in treating different human and livestock ailments and is widely employed for dental care. It has several names in accordance with the speaking population. In Arabic, it is commonly known as Miswak, Siwak, or Arak. Aranmakapicam is its name in the Indian language; this term translates to mustard tree or natural toothbrush in English. In Japan it is called Qesam, while in Latin, it is called mastic [10]. Generally, the word (Miswak or Siwak) in Arabic also indicates the action of rubbing the teeth for the purpose of cleaning using chewing sticks. This herb has a long history of over 7000 years of use by the Babylonian and Roman empires as a chewing stick; it was also used in the Greek empire [11]. In Islam, there has been a rise of a prophetic medicine that drives its practice from all actions and practices applied or recommended by the prophet Muhammad peace be upon him and it has been directed toward promoting health [12].

Due to the popular use of *S. persica* among Muslims, it was studied widely and is still under investigation in the hopes of discovering further unknown biological effects that might propose it as a new material of choice for certain medical interventions. The World Health Organization has recommended and encouraged the use of chewing sticks as an effective tool for oral hygiene in areas where such use is customary. In addition, *S. persica* has a long history of use as a medicine by many ethnic groups, particularly in Africa and Asia. All parts of the plant, including the flowers, fruits, leaves, bark, seeds, stems, and roots, have been used to treat many disorders related to various physiological systems in human beings including the circulatory, motor, excretory, and digestive systems [8].

*Salvadora persica* is classified into a kingdom called Plantae, a division called Magnoliophyta, a class called Magnoliopsida, a subclass called Dilleniidae, an order called Capparales, a family called Salvadoraceae, a genus called *Salvadora*, and a species called Persica. Usually, the part used as a cleaning stick is the root where the periphery would be cut, and the bristles are exposed for use as a toothbrush against teeth and the surrounding structure. The origin of *S. persica* can be considered a wide geographical distribution throughout the world in countries such as Saudi Arabia, Yemen, Iran, Iraq, Egypt, India, Pakistan, Malaysia, Sudan, Ethiopia, and Mauritania as well as countries in Central Africa, Southwestern Africa, and South America [6].

In term of its composition, all parts of *S. persica* have been screened. Extensive phytochemical analysis revealed the presence of carbohydrates, flavonoids, terpenes, sterols, alkaloids, and glycosides. Organic sulfur compounds and elemental sulfur were also present as small amounts of fluoride, calcium, phosphorus, silica, and ascorbic acid [8]. Another study found that the chemical constituents of *S. persica* were flavonoids, salvadorine, cyanogenic glycosides, lignans, saponins, alkaloids, tannins, linoleic acid, stearic acid, salvadourea, vitamin C, silica, and different salts, which was similar to the previous study [13]. Phytochemical screening of the aqueous extract of *S. persica* leaves revealed the presence of sterols/terpenes, flavonoids, flavone aglycone, saponins, and tannins. Furthermore, a study screened the extracts of *S. persica*'s twigs and stem using several extraction methods (hexane, chloroform, ethanol, and water extracts) for the presence of phytochemicals including alkaloids, glycosides, tannins, saponins, and flavonoids. All tested phytochemicals were absent in the hexane extract while only alkaloids were present in their chloroform extracts. In addition, the ethanolic extract contained all tested phytochemicals except for alkaloids and tannins. Finally, the aqueous extract contained all tested phytochemicals without alkaloids. These variations can be explained by the differences in solvent polarity to extract the phytochemical compounds from the plant [14]. On the other hand, another study observed tannin and saponin in the aqueous and ethanolic extracts, respectively [15]. The variations in extraction processes have been responsible for these varying results, which indicates that the importance of unifying and controlling the extraction methods.

Multiple biological effects of *S. persica* have been reported in the literature including antibacterial, antiviral, antifungal, antibiofilm, antioxidant, and even antiulcer effects. Detailed information will be presented. The purpose of this article is to narratively review the biological properties *of S. persica* and to present its various applications in different dental specialties.

## 2. *Salvadora persica* Biological Properties

### 2.1. Antibacterial Properties

Several in vitro studies have reported the antibacterial effects of Miswak on cariogenic bacteria and periodontal pathogens including *Staphylococcus aureus*, *Streptococcus mutans*, *Streptococcus faecalis*, *Streptococcus pyogenes*, *Lactobacillus acidophilus*, *Pseudomonas aeruginosa*, *Aggregatibacter actinomycetemcomitans*, and *Porphyromonas gingivalis*. Sher et al. [9] tested both aqueous and alcoholic extracts of *S. persica* against selected pathogenic microbes, *Staphylococcus aureus*, *S. mutans*, *Lactobacillus acifophilus*, and *Pseudomonas aeruginosa*, and concluded that aqueous extract showed significant inhibition in the growth of all pathogens tested with a profound inhibitory activity against *Staphylococcus* species compared to the alcoholic one. On the other hand, methyl alcohol extract had a significant antibacterial effect against *L. acifophilus* and *P. aeruginosa*. These results confirm the antibacterial effect, and further testing has been advocated. Investigations extended to explore the antibacterial effect of methanolic extracts on oral bacteria known to be associated with periodontitis concluded that *S. persica* was effective against most of the bacterial strains found in saliva [16]. Acetonic extract of *S. persica* had an inhibitory effect on the growth of nine isolated pathogenic bacteria of both human and plant with a much stronger effect on the latter [17]. The plant pathogens were *Agrobacterium tumefaciens*, *Pectobacterium atrosepticum*, *Enterobacter cloacae*, *Dickeya solani*, and *Ralstonia solanacearum*, while the human bacteria were *Bacillus subtilis*, *Sarcina lutea*, *Escherichia coli*, and *Staphylococcus aureus*. Interestingly, aqueous extract of *S. persica* showed strong antiprotozoal potential against the different subtypes of *Blastocystis* species in in vitro settings [18]. The natural antibacterial effect of *S. persica* has been confirmed and will always be of great interest to many medical and nonmedical specialties.

### 2.2. Antibiofilm Properties

The effect of *S. persica* against bacteria in planktonic format has been confirmed but bacteria usually live in a complex format called biofilm. It represents communities of bacteria attached to a surface and connected by a self-produced polymer matrix composed mainly of polysaccharides, secreted proteins, and extracellular DNA. Such complexity helps protect the bacteria and plays a crucial role in the chronicity of illnesses [19]. *S. persica* has shown promising antibiofilm effects. A study by Al-Sohaibani and Murugan [20] evaluated the inhibition and antibiofilm properties of methanolic, ethanolic, chloroformic, acetonic, and aqueoustic extracts of *S. persica* on *Streptococcus mutans* isolates. They evaluated the biofilm inhibition and concluded that the reduction percentages in biofilm for methanol, ethanol, chloroform, acetone, and aqueous extracts were 87.92%, 85.75%, 72.44%, 61.66%, and 58.68%, respectively. Also, their results indicated a dual antibiofilm function in the colonization and accumulation step besides its biofilm growth inhibition effect [20]. Khan et al. evaluated the antibiofilm and antimicrobial activity of fresh and dried roots of *S. persica* essential oils against *Streptococcus mutans*, then compared it to chlorhexidine digluconate (CHX) and clove oil using multiple assays. They concluded that essential oils demonstrated results comparable to that of CHX and showed a significant reduction in biofilm formation at a very low concentration. These results were supported by RT-PCR studies that showed changes in the expression of the AtlE, gtf B, ymcA, and sodA gene levels involved in autolysis, biofilm formation, and oxidative stress, respectively. These findings support the use of *S. persica* as an antibacterial product; further research should continue exploring it [21].

### 2.3. Antifungal Properties

Fungal infections are of great concern in dentistry. Patients may present with fungal infections that are indicative of a more serious systemic illness. The most prevalent fungal infection in the oral cavity is *Candida albicans* [22]. Several studies evaluated the biological effects of *S. persica* extracts on different types of fungal infections. For example, a study examined the antimicrobial effect of 20% *S. persica* extracts on *C. albicans* and *E. faecalis* using the dilution tube susceptibility test and confirmed the effectiveness of the extract against both species [23]. Balto et al. evaluated seven formats of *S. persica* extracts including hexane, chloroform, ethyl acetate, methanol-soluble, methanol-insoluble, ethanol, and water on the antimicrobial activity of *E. faecalis* and *C. albicans* by counting the colony-forming units (CFUs) at different periods and concluded that the hexane extract induced a steady and progressive significant reduction in CFUs for both *E. faecalis* and *C. albicans* at all concentrations and time periods. Similarly, significant progressive inhibition of *E. faecalis* CFUs was also observed for ethanol at all times, unlike the chloroform extract that showed this significance at 24 hours despite its concentration [24]. Another study tested the antifungal effects of solid and pulverized *S. persica* (which means grinding the substance into small parts) against multiple strains of oral *Candida* and confirmed the antifungal effect in both formats using the agar diffusion test. Interestingly, the volatile compounds in the solid format exhibited a strong growth inhibition effect unlike the pulverized format, which indicates that the storage as well as the size of the sticks affect growth inhibition [25]. Benzyl isothiocynanate (BITC), which is an active ingredient of *S. persica*, was also tested against *C. albicans* growth, cell size, morphogenesis, and ultrastructure effect. They investigated the antifungal potential of isothiocyanates (ITCs) against *C. albicans* oral isolates by a preliminary susceptibility disk diffusion test (DD) using allyl isothiocyanate (AITC), benzyl isothiocynanate (BITC), and phenyl ethyl isothiocyanate (PEITC), and concluded that aromatic ITCs have a strong inhibitory effect against *C. albicans*. In addition, the results suggest that BITC may be effectively used against *C. albicans* to modulate its growth and control or suppress its invasive potential [26]. Nevertheless, *S. persica* extracts were also potent against other types of fungus besides *C. Albicans*. Saddiq and Alkinani measured the antifungal suppressing effect of the aqueous extract of *S. persica* L. against three *Aspergillus* species (*A. niger*, *A flavus*, and *A fumigatus*) using radial growth rate and inhibition zone (IZO). Their results indicated a fungicidal effect of *S. persica* against aspergillosis [27].

### 2.4. Antioxidant Properties

The oxidative stress that is an imbalance in the oxygen radicals has been considered an issue affecting human health. This imbalance can lead to cell damage and have a negative impact on our health. Thus, the lack of antioxidants, which can promote reactive free radicals, might cause the development of degenerative diseases such as cardiovascular diseases, cancers, neurodegenerative diseases, Alzheimer's disease, and inflammatory diseases [28]. This aspect was explored with Miswak. A study evaluated variant *S. persica* crude extracts (methanol, ethanol, acetone, and water) for the presence of antioxidant molecules and concluded that the methanolic extract contained the highest amount of crude extract, which revealed high concentrations of antioxidant enzymes: peroxidase, catalase, and polyphenoloxidase. The synergistic action of antioxidative compounds and antioxidant enzymes makes Miswak a good chewing stick for cleaning teeth and improving oral hygiene [29]. Gupta et al. evaluated the antioxidant activity of chloroformic *S. persica* extract and compared it to the ethanolic extract [14]. They showed significant in vitro antioxidant activity in both extracts, but the chloroformic extract was more potent than the ethanolic one.

### 2.5. Anti-Inflammatory and Antiulcer Properties

Inflammation is a complex biological response of neurovascular tissues to harmful stimuli, such as pathogens, damaged cells, and irritants. It is an attempt to offer protection by clearing and removing the injurious stimuli to initiate healing. Interestingly, *S. persica* has an anti-inflammatory property as proven by Hoor et al., who induced inflammation in the hind paw of rats by subplanter injection of 0.1 ml of 1% carrageenan. The anti-inflammatory effect was measured by the volume of edema in the paw in milliliters using a plethysmometer, immediately before injection and then hourly up to five hours. The mean was then calculated. The researchers confirmed the *S. persica* anti-inflammatory effect on decreasing the paw volume of carrageenan-induced edema [30]. Moreover, studies explored the antiulcer effect of *S. persica*. Sanogo et al. studied the effect of *S. persica* administration prior to induced intragastric ulcers in rats and compared it to placebo. The results suggested that *S. persica* decoction possessed a significant protective action against ulcers induced by ethanol and by cold-restraint stress [31]. A recent study conducted by Lebda et al. evaluated the effects of *S. persica* aqueous extract on proinflammatory cytokines, nitric oxide synthases, apoptotic pathways, and oxidative/antioxidative pathways involved in ethanol-induced gastric ulcers in rats. They concluded that *S. persica* alleviated serious gastric mucosal ulcerations induced by ethanol and affirmed its efficacy as an antiulcer agent. The mechanism of action was believed to be through enhancing the antioxidative defense system, minimizing proinflammatory cytokines, upregulating apoptotic pathways, augmenting mucus content, and redesigning nitric oxide synthase (NOS) isoforms [32].

### 2.6. Cytotoxicity Properties

Cytotoxicity has always been an essential parameter for the biological evaluation of any material. The ideal antimicrobial agent mandates the microorganism's clearance while causing minimal toxicity to the host cells. Chemicals such as drugs and pesticides can be tested with in vitro settings to detect the mechanism of cytotoxic action, which can be through the destruction of cell membranes, the prevention of protein synthesis, irreversible binding to receptors [18]. The increasing interest in *S. persica* led researchers to study the cytotoxicity effects of the different *S. persica* extracts. Balto et al. assessed the potential cytotoxic effect of variant *Salvadora persica* extracts on human gingival fibroblasts. They used hexane, ethylacetate, and ethanol at 0.5 and 1 mg/ml concentrations. The study concluded that the ethanol and hexane extracts of *S. persica* at both concentrations were completely devoid of cytotoxic activity. In fact, hexane extract showed slight cytotoxicity compared to controls, but it was still considered low. The rest of the extracts showed more cytotoxic effects [33]. Sardari et al. evaluated the cytotoxic effect of Miswak on human oral Jurkat (T leukemia) cells which were an immortalized line of human T lymphocyte cells that can be used to study acute T cell leukemia, T cell signaling, and the expression of various chemokine receptors. The water extraction method from Miswak was used and tested at different concentrations for the cytotoxic and anti-inflammatory activities. The results suggested that *S. persica* caused a dose-dependent decrease in IL-6 and IL-8 secretion. It was confirmed that the stick extract exerted more cytotoxic effects on Jurkat cells than the leaf extract of the same *S. persica* herb [34]. Cancerous cells have been tested with *S. persica* as in Hammad et al., who examined the herbal effect on oral epithelial dysplasia cells (DOK), oral squamous cell carcinoma (PE/CA-PJ15), and periodontal ligament fibroblast (PDL) cell lines. Aqueous extracts of *S. persica* were used in high concentrations in this study; then, the cellular survival and proliferation effect was determined using the MTT assay, while the apoptotic effect was evaluated by Hoechst stain. The researchers concluded that the aqueous root extract of *S. persica* produces cytotoxic effects at lower concentrations in DOK and oral squamous cell carcinoma cells than in normal PDL cell lines. The overall results of the study suggest a potential role of S. persica in cancer prevention [35]. In addition, Al Bratty et al. evaluated the cytotoxic and antimicrobial properties of the *S. persica* fruit extract against three cancer cell lines: MCF7 (human breast carcinoma cells), A2780 (human ovary carcinoma cells), and HT29 (human colon carcinoma cells) and on MRC5 (normal human fibroblast) cells. They concluded that the ethanol extract showed good cytotoxic properties against ovary and colon cancer cells and lesser cytotoxicity against MRC5 normal cells. The results also suggest antimicrobial activity against *Streptococcus mutans* that was resistant to the standard drug ampicillin. These interesting findings confirm the anticarcinogenic and antimicrobial activity of *S. persica* and advocate for the extraction of *S. persica* from fruits and not only sticks and leaves [36]. Moreover, ethanolic and water extracts of *S. persica* in different concentrations were evaluated regarding the proliferation and viability of human dental pulp stem cells (hDPSCs). The studied concentrations of both extracts ranged from 5.75 mg/ml to 0.08 mg/ml and were tested using the MTT assay. The results indicated that methanolic extracts showed severe cytotoxicity in all concentrations except 0.71 mg/ml to 0.08 mg/ml, which are the lowest concentrations tested. Water extracts showed cytotoxic effect only at the highest concentration tested, which was 5.75 mg/ml [37].

## 3. Dental Applications of *Salvadora persica*

Dental caries is the most prevalent dental disease and has been one of the most concerning diseases among all humans. The origin of caries is bacteria and their byproducts, which cause a breakdown of the teeth and the surrounding gingival tissues, leading to pulpal and periapical diseases [38]. Dental plaque is an example of a biofilm that has a primary role in the pathogenesis of such a disease; it naturally develops on tooth surfaces [39]. The causative role of this biofilm in oral diseases lies mainly in adhesion, biofilm development, and resistance [22]. Maintaining good oral hygiene by chemical and mechanical means can help prevent microflora from accumulating and causing disease. As a part of the chemical means, multiple reports have studied the effect of *S. persica* on oral bacteria and plaque to evaluate the use of this material in all dental specialties. A study was conducted to evaluate the antibacterial activity of ethanolic and methanolic *S. persica* extracts against isolated genetically identified oral cavity pathogens from saliva using PCR amplifications, which were *Staphylococcus aureus* strain, *Enterococcus faecalis* strain, and *Klebsiella pneumoniae* strain. The study concluded that all *S. persica* extracts showed powerful antimicrobial activity against the mentioned pathogens. Moreover, the methanolic extract showed the highest inhibition against *E. faecalis*, while showing the lowest inhibition against *K. pneumoniae* [40]. Other studies have been conducted to evaluate *S. persica*'s role within different dental specialties.

### 3.1. Periodontics

There is great interest in studying Miswak in the field of periodontics. Two main microbial species causing destructive periodontal disease (*Aggregatibacter actinomycetemcomitans* and *Porphyromonas gingivalis*) have been tested with *S. persica* to assess the plant's antimicrobial activity. Plaque samples from patients with moderate to severe periodontitis were gathered from the deep periodontal pockets. Interestingly, *S. persica* had significant antimicrobial activity against *P. gingivalis* but not against *A. actinomycetemcomitans* as compared to 0.2% chlorhexidine [41]. Moreover, other forms of *S. persica* were tested as in Amoian et al. in 2010, who aimed to evaluate the effect on periodontal health of a chewing gum containing *S. persica*. The plaque index, gingival index, and bleeding index were all measured and followed for up to 14 days. There was a statistically significant reduction in the gingival index and bleeding index but not in the plaque index [42]. In addition, the plaque removal effect of gel form *S. persica* was studied and compared to photoactivated disinfection (PAD) in experimentally induced gingivitis. The plaque index and bleeding index were assessed and the microbiological parameter counts of five periodontal pathogens were evaluated. The results concluded that both PAD and *S. persica* gel improved plaque index. However, PAD reduced more bacterial counts while *S. persica* gel had a significant impact on the bleeding index [43]. *S. persica* also showed its effectiveness when used as a mechanical tool to remove plaque. In a recent meta-analysis conducted by Adam et al., where they aimed to find an answer as to whether *S. persica* brushing had an impact on the plaque and bleeding scores of healthy individuals compared to a standard toothbrush. They concluded that the persica chewing stick was a comparable tool for plaque control compared to a standard toothbrush and had a better antigingivitis effect [44]. Another important aspect of maintaining good periodontal health is mouth rinses. *S. persica* mouthwash was proven to significantly reduce plaque scores and bacterial counts compared to chlorhexidine according to a meta-analysis conducted in 2019 [45]. Nevertheless, *S. persica* was also tested in combination with 4 types of antibiotics to assess its synergistic antibacterial efficacy on selected periodontal pathogens. Ethanolic *S. persica* was assessed and plaque samples were collected from periodontitis patients for isolate pathogens (*P. gingivalis*, *T. denticola*, *T. forsythia*, and *A. actinomycetemcomitans*). The researchers concluded that the synergistic test showed significant antibacterial activity when plant extract was combined with an antibiotic. Specifically, a synergism effect was exhibited between *S. persica* with metronidazole against *A. actinomycetemcomitans* and *S. persica* with tetracycline against *P. gingivalis*, *T. denticola*, and *T. forsythia* [46]. In periodontics, the focus is on not only curing the diseased periodontal tissues, but also healing and repairing them. A study was conducted to compare the effects of chlorhexidine and *S. persica* on alveolar bone healing following tooth extraction in rats. The rats were mouth-rinsed for 2 weeks and extraction of the right mandibular molars was carried out after 8 days. The inflammatory cells in the extraction site were recorded after the rats were sacrificed. The results showed no significant difference in new bone formation and inflammatory cell counts between the two groups. However, mean bone formation was significantly higher in the *S. persica* group compared to chlorhexidine and the extraction socked wound healing was also more enhanced [47].

### 3.2. Restorative

It is of the utmost importance to maintain the health of natural dentition by understanding teeth composition and how to protect it. Also, it is important to restore the function, health, and integrity of a defective tooth structure when teeth are carious or traumatized. To do so, restorative materials are used and must be biocompatible, as well as have a good sealing ability while withstanding occlusal forces [48]. Multiple materials have been applied, starting with gold and amalgam restoration and ending with photo- and chemical-activated restorations such as composite and glass ionomer cements (GICs). However, these materials are still not considered ideal due to drawbacks such as shrinkage and the risk of microleakage [49]. For these reasons, studies to improve the properties of restorative materials have recently been of interest. Miswak showed its effectiveness in enhancing the properties of restorative materials such as glass ionomer cement (GIC) as proven by El-Tatari et al., who investigated the physical and antimicrobial properties of GIC when combined with ethanolic *S. persica* extracts at 3 different concentrations. The *S. persica* extracts were added to GIC; then compressive and tensile strengths were measured. Antimicrobial effects were also evaluated with specific microorganisms. The results showed that 4% of *S. persica* showed weaker strength compared to control, while 1% and 2% showed similar results to control. Regarding antimicrobial effects, specimens containing *S. persica* showed a significant increase in inhibition to microorganisms compared to pure GIC [50]. Moreover, alcoholic extraction of *S. persica* was tested in three different concentrations and was combined with GIC; then, compressive strength and antimicrobial activity were tested in comparison to chlorohexidine-modified GIC. The results revealed that the plant extracts enhanced the antimicrobial activity, especially against *S. mutans*. Meanwhile, the compressive strength was improved by the addition of the plant extracts in higher concentrations [51]. The inhibitory effect of *S. persica* on the collagen degradation of a demineralized dentin lesion was also studied. Aqueous extraction of *S. persica* was evaluated against demineralized bovine root dentin specimens for 3 days, and then viewed by using a light microscope. The results showed that the extract preserved the dentin collagen matrix from the collagenase enzyme, which suggests that *S. persica* might have a positive effect in caries prevention [52].

### 3.3. Endodontics

The main objective of endodontic treatment is to maintain and preserve the health of pulpal and periapical tissue. The cause of endodontic disease, whether it is a primary disease or post-treatment infection, has been proven throughout years of study to be bacteria [38]. However, the microbes in infected root canals can be much more complicated to treat, especially when they are in multispecies microbial communities, which are known as biofilm [53]. The success of endodontic treatment relies on the combination of chemical and mechanical instrumentation to disinfect the root canal system, followed by canal obturation to prevent the reentry of bacteria and their byproducts [54]. However, in failed cases or post-treatment disease, multiple facultative anaerobic bacteria have been proved to be the cause. One of the most detected microorganisms in persistent endodontic infections is *Enterococcus faecalis* (*E. faecalis*) [55]. For this reason, *S. persica* was evaluated against endodontic pathogen isolates from teeth with failed RCT. The study used *S. persica* along with other plant extracts in combination with different antimicrobial agents such as penicillin and tetracycline against different endodontic pathogens including *E. faecalis*. The results indicated the effectiveness of *S. persica* in combination with the abovementioned antimicrobial agents against all experimental pathogens except *Candida albicans* [56]. Irrigation solutions such as sodium hypochlorite and chlorhexidine are considered a form of chemical control of the infected canals. *S. persica* was applied in multiple studies as either an endodontic irrigant or even an additive to sealers. For example, Devi et al., in 2019, evaluated and compared the antimicrobial efficacy of root canals sealers using different bases. *S. persica* was mixed with three types of endodontic sealers along with other herbal products and the mean zones of inhibition for nine strains of bacteria were measured. They concluded that *S. persica* mixed with either AH+ or Apexit plus showed the second and third largest zones of bacterial growth inhibition [57]. As for irrigation, *S. persica* did not show the best antibacterial efficacy as compared to *Hymus vulgaris, Acacia nilotica, Calendula arvensis*, and 5% sodium hypochlorite against *E. faecalis* [58]. However, *S. persica* showed fewer changes in the microhardness of root dentin when used as an irrigant compared to 2.5% NaOCl [59]. In addition, the efficacy of *S. persica* was evaluated in the elimination of the intracanal smear layer. In a study aimed at comparing ethanolic *S. persica* extract to 17% EDTA using scanning electron microscopy (SEM), *S. persica* solution was as effective as 17% EDTA in removing the smear layer from the coronal third of the canal wall [60]. Although multiple studies mentioned the use of *S. persica* in endodontics, the biological activity of this plant is still a wide space for investigation and future implementation, whether as an additive to material or used itself.

### 3.4. Pediatrics and Orthodontics

It is believed that the oral health of a child mirrors that child's general health and is a strong predictor of oral health in adulthood. Therefore, it is important to understand oral health and disease, including periodontal tissue, to promote longstanding oral health [61]. For this reason, *S. persica* was studied to evaluate the antimicrobial activity of methanolic extracts on the oral health of children presented with decay. The study was conducted in vitro and in vivo by collecting plaque samples from selected children to evaluate the antibacterial properties and administration of *S. persica* mouthwash and compare this group to a placebo. The results showed a statistically significant difference in colonization levels using *S. persica*, especially Gram-negative bacteria. The in vitro study revealed a significant reduction in bacteria of the oral cavity using *S. persica* mouthwash as compared to placebo [62]. Moreover, a randomized double-blinded clinical trial was conducted and aimed to evaluate the effect of *S. persica* brushes on the count of *Streptococcus mutans* and the mean plaque score in children. The sample included high caries-risk children who were subjected to either an *S. persica* brush or a regular soft brush. The researchers concluded that the *S. persica* brush along with fluoridated toothpaste significantly reduced plaque levels compared to a regular toothbrush and that the proportions of salivary bacteria also changed, with less risk of inducing caries [63]. In orthodontic patients, the oral environment undergoes several changes including retention sites that increase the accumulation of food particles, eventually causing decalcification lesions. For this, *S. persica* in hexane and ethanol extract methods was applied on a monospecies biofilm model established on orthodontic brackets to evaluate the antimicrobial potential. The study was conducted in vitro, and the bacterial cell viability of the biofilm was measured after exposure to both *S. persica* extracts compared to chlorhexidine and saline. The results revealed that hexane *S. persica* extract showed a decline in the bacterial cell viability of *S. mutans* and was more effective than ethanolic extract and nearly as effective as chlorohexidine. This suggests the potential use of *S. persica* extracts as an oral antimicrobial agent for orthodontic patients [64].

## 4. Conclusion

This review expresses narratively the biological effects of *Salvadora persica* and some confirmed effects in different dental specialities. It is a promising agent that can have a wider range of benefits beyond those of which we are currently aware. Based on its properties, future applications in regenerative dental treatments seem reasonable.

## Data Availability

The data are available on request.
